# Exercise-Diet Therapy Combined with Insulin Aspart Injection for the Treatment of Gestational Diabetes Mellitus: A Study on Clinical Effect and Its Impact

**DOI:** 10.1155/2022/4882061

**Published:** 2022-07-28

**Authors:** Amei Mu, Yan'e Chen, Yongmei Lv, Wenxing Wang

**Affiliations:** ^1^Interventional Department of Nephrology, The Affiliated Qingdao Central Hospital of Qingdao University, The Second Affiliated Hospital of Medical College of Qingdao University, Qingdao 266042, China; ^2^Department of Neurology IV, Jiyang People's Hospital, Jinan 251400, China; ^3^Department of Pharmacy, Zhangqiu District People's Hospital, Jinan 250200, China; ^4^Department of Obstetrics I, Yantaishan Hospital, Yantai 264000, China

## Abstract

**Objective:**

To explore the clinical effect and impact of exercise-diet therapy combined with Insulin Aspart Injection on gestational diabetes mellitus (GDM).

**Methods:**

The objects of study were patients with pregestational diabetes mellitus (PGDM) and 62 patients with GDM who were diagnosed by oral glucose tolerance test (OGTT) and insulin release test from February 2017 to February 2019. According to the severity of the disease, enrolled patients were informed to have appropriate exercise and diet control or Insulin Aspart Injection on this basis until the completion of delivery. By using 50 pregnant women with normal glucose as the control, the fasting plasma glucose (FPG), 1-hour postprandial glucose (1hPG), 2-hour postprandial glucose (2hPG), nocturnal glucose, and glycosylated hemoglobin (HbA1c) levels were compared between the PGDM group and the GDM group before and after treatment; besides, further comparison was made in terms of glucose compliance rate, islet B-cell secretory function, and insulin resistance after treatment. The pregnant women were examined by B-ultrasound at 24 and 26 weeks of gestation to check if the fetus had abnormalities in the central nervous system and the heart. Further B-ultrasound examination was performed at 32 and 37 weeks of gestation to check the problems such as polyhydramnios and stillbirth. In addition, a comparative analysis was carried out in terms of the adverse pregnancy outcomes and complications, associated with the comparison of the results after treatment with control group.

**Results:**

After treatment, the levels of FPG, 1hPG, 2hPG, nocturnal glucose, and HbA1c were decreased in the PGDM group and GDM group than those before treatment, especially in the GDM group, with significant difference still when compared with the control group (*P* < 0.05). Statistical analysis revealed that the blood glucose compliance rate in the GDM group was higher than that in the PGDM group, showing a better therapeutic effect. Fasting insulin (FINS) and homeostasis model assessment index for insulin resistance (HOMA-IR) in the GDM group were significantly higher than those in control group, but lower than those in the PGDM group (*P* < 0.01), while the level of HOMA-*β* was lower in the GDM group than that in the control group and higher than that in PGDM (*P* < 0.01). Further ultrasound examination revealed the presence of fetal cardiac abnormality, polyhydramnios, stillbirth, and problems, showing a higher incidence in the PGDM group but almost nonexistence in the control group. In addition, the incidence of hypertension, macrosomia, premature rupture of membranes, postpartum hemorrhage, and infection were obviously higher in the PGDM group than those in the GDM group and control group (*P* < 0.05).

**Conclusion:**

Exercise-diet therapy combined with Insulin Aspart Injection can effectively control the blood glucose level of pregnant patients with GDM, improve the pregnancy outcome to a certain extent, and ensure the health of pregnant women and fetus, which is worthy of clinical application.

## 1. Introduction

Diabetes mellitus is a type of metabolic disease characterized by high blood glucose, with insulin secretion defect or biological damage acting as its major reason of pathogenesis. The diagnostic criteria for hyperglycemia during pregnancy was revised by the Chinese Diabetes Society (CDS) in the 2016 Guidelines [1]. Pregnancy associated with diabetes mellitus can be divided into the following two types, diabetes mellitus patients getting pregnant (pregestational diabetes mellitus, PGDM) and pregnant patients with diabetes mellitus (gestational diabetes mellitus, GDM). According to previous research [2–4], about 1%~15% of pregnant women have GDM annually. It can be explained by the impact of pregnancy that may change the immune system and endocrine system of females, resulting in increased demand for glucose, insufficient insulin secretion, or insulin resistance and hence increasing the risk of diabetes mellitus. It is well known that hyperglycemia during pregnancy has an intimate association with maternal, fetal, and neonatal morbidity. Diabetes mellitus is a high-risk factor for adverse pregnancy outcomes and complications. For instance, compared with pregnant women with normal blood glucose, patients with diabetes mellitus have higher risk to develop fetal intrauterine dysplasia, neonatal malformation, macrosomia, and other symptoms, while the mothers are prone to have preeclampsia and develop into type 2 diabetes mellitus after delivery in the case of poor control. Therefore, the risk of adverse pregnancy outcomes of GDM patients is significantly higher than that of pregnant women with normal blood glucose, and that of PGDM patients is higher than that of GDM, which has been concerned greatly in recent decades. In this regard, there is a need to pay much attention to the nursing methods in order to ensure the health and safety of pregnant women and newborns.

It has been reported that the application of medical intervention to patients with diabetes mellitus can greatly reduce the probability of perinatal diseases, ensure women's health, improve their related quality of life, and reduce the risk of birth of unhealthy fetuses and dystocia [5]. It is thus necessary for patients with gestational hyperglycemia to receive appropriate treatment. However, according to different medical conditions of patients and treatment goals, still 10%-30% of patients with gestational hyperglycemia require medical treatment on the basis of lifestyle intervention [6]. Insulin is the preferred choice for treating patients with hyperglycemia [7, 8]. While in view of the advantages of oral hypoglycemic drugs in cost and convenient use, it has aroused great interest in the treatment of gestational hyperglycemia recently. Comparison on the safety and effectiveness of oral hypoglycemic drugs with insulin and insulin analogues has become the major focus of the current concern in the treatment of gestational hyperglycemia. For example, existed systematic analysis on the treatment of GDM with insulin has compared and analyzed the safety and effectiveness between insulin and oral hypoglycemic drugs. Corresponding results revealed that insulin and oral hypoglycemic agents produced similar efficacy in major health outcomes. At present, insulin is the first choice for the treatment of gestational diabetes mellitus, as an effective drug for blood glucose control. Accordingly, the present study was conducted to explore the clinical effect and adverse pregnancy outcomes of Insulin Aspart Injection combined with exercise-diet therapy in the treatment of GDM, and the report is as follows.

## 2. Materials and Methods

### 2.1. General Data

The objects of study were 55 patients with PGDM and 62 patients with GDM (*n* = 117 in total) diagnosed in our hospital from February 2017 to February 2019 according to the *Guidelines for the Diagnosis of Gestational Diabetes Mellitus (2016 Edition)* [9]. According to the severity of disease, all patients were treated with appropriate exercise, diet control, and intensive therapy with Insulin Aspart Injection during hospitalization. The control group was pregnant women with normal blood glucose level (*n* = 50). The exclusion criteria were subjects with severe infection; genetic disease; failure of important organs; endocrine disease; refusal of drug therapy; allergy to the medicine used in this study; and acute complications such as diabetic ketoacidosis, damage in the heart, liver and kidney, hyperthyroidism, pancreatitis, anemia, and other diseases affecting blood glucose level [10]. This study obtained approval from the Ethics Committee of our hospital, following the principle of the Declaration of Helsinki (as revised in 2013). The patients have signed informed consent.  Table 1 shows the general data of enrolled subjects.

### 2.2. Therapeutic Methods [11–14]

The therapeutic methods were described in detail as follows: the diet style of patients was having more meals a day but less food at each, with attention paid to avoid foods with high sugar content, reduce the amount of staple food, and increase the proportion of coarse food grains as the best choice. It was recommended to strengthen appropriate exercise after three meals (such as walking for 15-30 minutes) and keep individualized diet and some exercise support. Basic insulin should be injected at bedtime every day, and Insulin Aspart should be injected before three meals (NovoRapid, Novo Nordisk China Pharmaceutical, National medicine approval No. J20100124, 3 ml: 300 IU). The dosage was adjusted to 0.5-1.0 IU/kg/d according to the severity of the patient's condition and the monitoring results of blood glucose. The treatment was continued until delivery. The method of blood glucose level monitoring was as follows: (1) blood glucose monitoring. Patients were instructed to measure the blood glucose individually and use the blood glucose meter regularly. The blood glucose level is directly proportional to the incidence of complications in pregnant women and fetuses. Hence, the fluctuation of blood glucose must be monitored in a strict manner to provide an effective basis for subsequent treatment. (2) Medication instruction. The correct method of Insulin Aspart Injection and the working mechanism of insulin were explained in detail in stages, so as to cultivate the consciousness of patients to measure blood glucose voluntarily and form the habit gradually. It was expected to ensure that patients could understand the adverse reactions and possible results of drugs fully and enhance their awareness of the standard medication. (3) Diet care. According to the individual blood glucose level, patients were guided to strictly control the total calorie intake of food daily, so as to better control the blood glucose; besides, based on the dietary habit and preference, patients were informed to choose the type of food for regular and quantitative intake, and spare a certain space; patients could select favorite food in a certain range, improve their compliance behavior as much as possible, but do not increase or reduce the amount of food unadvisedly. Meanwhile, patients should have more food with high cellulose, supplement some fresh fruits and food containing trace elements needed by the human body, and prohibit spicy, raw, and cold food with high sugar and large amount of oil, so as to ensure a light diet in the daily life. (4) Excise care. Patients were instructed to take exercise 1 hour after meal for 30 min/time each time and pay attention to have moderate exercise to experience the feeling of a little weak and slight sweating after exercise and comfortable feel after rest. It was recommended to avoid strenuous exercise, fasting excise, excise when there was physical discomfort, and excise during the waiting time for meals after insulin injection and have exercise safely to prevent falling to induce abortion. Proper exercise may be beneficial to maintain the health of pregnant women and fetus, better control of blood glucose, reduce patients' demand for insulin, and improve glucose tolerance.

### 2.3. Diagnostic Criteria

According to the recommended criteria mentioned in the *Guidelines for the Diagnosis of Gestational Diabetes Mellitus (2016 Edition)*, 75 g OGTT was used to measure blood glucose at 24-28 weeks and on the first visit after 28 weeks of gestation. Patients were confirmed with GDM when any of the blood glucose values reached or exceeded the above criteria: PG5: 1~6.9 mmol/L, blood glucose ≥ 10.0 mmol/L 1 h after OGTT, and blood glucose ≥ 8.5 and <11 mmol/L 2 h after OGTT. Besides, PGDM was diagnosed in patients with definite history of diabetes mellitus before pregnancy.

### 2.4. Observational Indexes

Blood glucose indexes, including fasting blood glucose (FPG), 1-hour postprandial glucose (1hPG), 2-hour postprandial glucose (2hPG), and nocturnal glucose and glycosylated hemoglobin (HbA1c) levels, were recorded before and after treatment. In terms of the major observational indexes, the blood glucose control of gestational hyperglycemia was performed in accordance with the standard recommended by the *Guidelines for the Diagnosis of Gestational Diabetes Mellitus (2016 Edition)*. FPG should be controlled between 3.3~5.3 mmol/L, 2hPG ≤ 6.7 mmol/L, 1hPG ≤ 7.8 mmol/L, and nocturnal blood glucose > 3.3 mmol/L, and HbA1c during pregnancy should be <5.5%. Moreover, the secretory function of islet-B-cells and insulin resistance-related indexes were recorded [6, 15], associated with the detection of fasting insulin (FINS). Furthermore, islet B-cell secretion index (HOMA-*β*) and homeostasis model assessment index for insulin resistance (HOMA-IR) were used to evaluate islet B-cell secretory function and insulin resistance, of which HOMA − *β* = FINS × 20/(FPG − 35); HOMA − IR = FPG × FINS/22.5. Simultaneously, the adverse pregnancy outcomes were analyzed, including polyhydramnios, macrosomia, postpartum hemorrhage, and postpartum infection. In this study, blood glucose was measured 4-7 times a day, and it was controlled in the above range by combining the intensive therapy of Insulin Aspart Injection. The experiment was repeated three times.

### 2.5. Use of Instruments

The instrument for measuring peripheral blood glucose used BaiAnJin blood glucose meter (7600P, Bayer HealthCare LLC.). Other instruments included ion-exchange high-performance liquid chromatography (BIO RAD VARIANT II, Bio-Rad Laboratories, Inc., USA) and glycosylated albumin monitoring kit (Abbott I16200, Abbott, USA).

### 2.6. Statistical Analysis [16]

The SPSS 23.0 statistical software was used to analyze and process the data in this study. The count data (%) were tested by *χ*^2^ test, and the measurement data (*x̅*±*s*) were examined by *t*-test. *P* < 0.05 meant that the difference was statistically significant.

## 3. Results

### 3.1. Comparison of Blood Glucose Index and Blood Glucose Compliance Rate

Measurement results were compared according to the blood glucose control criteria in the *Guidelines for the Diagnosis of Gestational Diabetes Mellitus (2016 Edition)*. As shown in Table 2, after reasonable treatment, levels of FPG, 1hPG, 2hPG, nocturnal glucose, and HbA1c were decreased in the PGDM group and GDM group than those before treatment, especially in the GDM group when compared with the PGDM group, with significant difference still when compared with the control group, with statistical significance (*P* < 0.05). Further analysis of the blood glucose compliance and calculation of corresponding rate [17] showed that the rate was much higher in GDM (Figure 1), exhibiting better therapeutic effect.

### 3.2. Comparison of Islet-B-Cell Secretory Function and Insulin Resistance-Related Indexes among Groups

After treatment, FINS and HOMA-IR in the GDM group and PGDM group decreased significantly [18], which were better in the control group when compared with combined diabetes mellitus group, while HOMA-*β* was increased in the GDM group and PGDM group, which was the highest in the control group (Table 3).

### 3.3. Monitoring of the Unborn Fetal Health

According to the results of B-ultrasound [19, 20] of pregnant women in the second and third trimester, the fetal health of the GDM group was better than that of the PGDM group after treatment, and there was almost no adverse reaction in the control group (Figure 2).

### 3.4. Comparison of Adverse Outcomes and Complications of Pregnant Women

As shown in Table 4, after treatment, the adverse pregnancy outcomes and complications of the GDM group were better than those of the PGDM group (*P* < 0.05); comparison among groups showed that the control group had a better adverse pregnancy outcomes and complications.

## 4. Discussion

The incidence rate of pregnancy combined with diabetes mellitus [21] is as high as 17.5% in China. It includes two types, as described below. In the first type, subjects have got diabetes mellitus before pregnancy in the absence of blood glucose test, which is known as PGDM; as for the second type, there is no abnormality in the level of blood glucose before pregnancy, while the internal hormone changes due to the special physiological reaction of pregnant women during pregnancy, resulting in impaired glucose tolerance and diabetes mellitus, which is called GDM. In general, diabetes mellitus may produce variety of perinatal complications that may have a great impact on the development of pregnant women, fetuses, and newborns [22, 23]. The absence of timely and effective control of blood glucose of pregnant women, the mother, and baby during the prenatal period may develop various serious complications and even death. It has been documented that several important factors can lead to the occurrence of GDM, such as obesity, old age, family history of diabetes mellitus, and poor birth history [24]. In addition, emotional, psychological, and physiological guidance for women with GDM are of great significance in reducing the incidence of complications and improving pregnancy outcomes.

There exists a cause-effect relationship between pregnancy and diabetes mellitus in GDM. Pregnancy may result in the domination of diabetes mellitus and may also lead to the aggravation of hyperglycemia in pregnant women. Diet therapy, exercise therapy, and insulin therapy are all available choice for the treatment of GDM in the clinical setting [25]. In the mild stage, diet therapy combined with moderate exercise therapy may play a therapeutic effect on controlling the blood glucose effectively, while for patients with moderate and severe conditions, there is a need to apply intensive therapy using insulin. During pregnancy, pregnant women may experience extremely obvious increase in estrogen and progesterone secretion. It may further increase insulin secretion, cause antagonistic effect, and finally generate insulin resistance, resulting in abnormal blood glucose level of pregnant women [26]. At present, HOMA-IR has been recognized to be the most commonly used index to evaluate the degree of insulin resistance. In our study, there was a significantly higher level of HOMA-IR in the PGDM group and GDM group than that in the control group, suggesting a more obvious insulin resistance in patients with diabetes mellitus. Furthermore, following the decrease of insulin sensitivity and the increase of insulin resistance, for the purpose of regulating the blood glucose level, the function of islet B-cells may exhibit a compensatory enhancement to maintain the blood glucose within the normal range. It may consequently show an enhanced secretion of islet B-cells. Nevertheless, in the case of excessive enhancement in insulin resistance, the blood glucose may increase when the insulin secreted by islet B-cells is not enough to compensate. As revealed in our study, HOMA-*β* was evidently lower while FINS was much higher in the PGDM group and GDM group than those in the control group. The insufficient islet secretion in patients combined with diabetes mellitus may be attributed to the deficiency of primary B-cell secretion. In addition, high blood glucose can inhibit the secretion of islet B-cells, which can also suppress the secretion ability of islet B-cells, and even cause permanent damage to islet B-cells. Consequently, the insufficient insulin secretion may further increase blood glucose, which will eventually aggravate insulin resistance repeatedly, forming a vicious circle. Insulin Aspart [27, 28] is a common choice in the medicinal treatment of GDM. Our study carried out a comparative analysis concerning the effect of Insulin Aspart Injection on patients with PGDM and GDM. Corresponding results indicated a certain decrease in the blood glucose index and adverse pregnancy outcome in both groups. It may suggest that Insulin Aspart Injection can achieve an effective control on the blood glucose level, regulate oxidative stress state of patients, and consequently ensure the safety of pregnant women, fetus, and newborn. In accordance with the aforementioned interpretation, it can be found that Insulin Aspart can exert the hypoglycemic effect of insulin, and its activity is close to that of natural insulin. It has rapid work and absorption and can reach the peak of plasma concentration quickly, with relatively short half-life.

To sum up, GDM patients may experience obvious compensatory insufficient insulin secretion and insulin resistance, as well as high risk of adverse pregnancy outcomes compared with pregnant women with normal blood glucose. Therefore, once GDM is diagnosed during pregnancy, it is recommended to actively adopt a series of interventions such as drugs and diet. The exercise-diet therapy combined with Insulin Aspart Injection applied in our study can improve the pregnancy outcome of patients with GDM, effectively control blood glucose, and improve maternal and neonatal complications.

## Figures and Tables

**Figure 1:** The blood glucose compliance rate (%) of the PGDM group and GDM group after treatment.

**Figure 2:** Monitoring of the unborn fetal health. (a) A 30-year-old PGDM patient with intrauterine pregnancy. (b) A 28-year-old GDM patient with intrauterine pregnancy. (c) A 31-year-old PGDM patient with single fetus.

**Table 1:** General data of enrolled subjects (*x̅*±*s*).

Items	PGDM group	GDM group	Control group	*χ* ^2^	*P*
Cases	55	62	50		
Age (year)	29.54 ± 4.31	28.71 ± 4.73	29.37 ± 5.07	0.352	>0.05
Weight (kg)	78.8 ± 11.3	76.2 ± 13.2	78.1 ± 12.5	1.247	
Gestational age (week)	25.75 ± 3.50	28.50 ± 5.25	27.25 ± 3.75	4.833	
Gravidity and parity (times)	1.17 ± 0.33	1.06 ± 0.23	1.12 ± 0.26	0.113	
With family history of disease	26 (47.3)	11 (17.7)	-	0.638	
HbA1c (%)	16.3 ± 2.5	15.6 ± 1.7	4.8 ± 0.34	8.576	

PGDM: pregestational diabetes mellitus; GDM: gestational diabetes mellitus; FINS: fasting insulin.

**Table 2:** Blood glucose index (*x̅*±*s*) and blood glucose compliance rate (%).

Group	Time	Case	FPG (mmol/L)	1hPG (mmol/L)	2hPG (mmol/L)	Nocturnal glucose (mmol/L)	HbAlc (%)
PGDM group	Before treatment	55	6.83 ± 0.46	11.27 ± 1.94	9.84 ± 1.23	5.71 ± 0.22	7.7 ± 0.6
	After treatment		5.61 ± 0.37^a^	8.06 ± 0.47^a^	7.08 ± 0.42^a^	4.65 ± 0.28^a^	6.1 ± 0.7^a^
GDM group	Before treatment	62	6.62 ± 0.33	11.66 ± 1.64	9.76 ± 1.27	5.57 ± 0.24	7.2 ± 0.4
	After treatment		5.15 ± 0.34^a^	7.57 ± 0.32^a^	6.54 ± 0.39^a^	4.04 ± 0.26^a^	5.3 ± 0.4^a^
Control group		50	4.06 ± 0.21	7.13 ± 0.26	5.73 ± 0.34	3.86 ± 0.23	4.7 ± 0.3
*P*			<0.05^∗^	<0.05^∗^	<0.05^∗^	<0.05^∗^	<0.05^∗^

**Table 3:** Comparison of islet-B-cell secretory function and insulin resistance-related indexes among groups (*x̅*±*s*).

Group	Time	Cases	FINS (mU/L)	HOMA-*β* (%)	HOMA-IR
PGDM group	Before treatment	55	37.13 ± 5.47	5.18 ± 0.21	3.64 ± 1.13
	After treatment		12.31 ± 2.56^a^	7.03 ± 0.41^a^	2.93 ± 0.66^a^
GDM group	Before treatment	62	36.75 ± 6.38	5.68 ± 0.24	3.58 ± 1.27
	After treatment		6.64 ± 1.75^a^	8.36 ± 0.37^a^	2.31 ± 0.35^a^
Control group		50	2.41 ± 1.03	9.22 ± 0.15	1.72 ± 0.12
*χ* ^2^			14.537	6.263	4.712
*P*			<0.05^∗^	<0.05^∗^	<0.05^∗^

Note: PGDM: pregestational diabetes mellitus; GDM: gestational diabetes mellitus. Compared with pretreatment condition, *P*^a^ < 0.01. Comparison between the PGDM group and the GDM group, *P* < 0.01. Compared with the control group, *P* < 0.01.

**Table 4:** Comparison of adverse outcomes and complications of pregnant women (*n*(%)).

Group	Cases	Hypertension	Premature rupture of membranes	Macrosomia	Postpartum hemorrhage	Postpartum infection
PGDM group	55	10 (18.2)	8 (14.5)	6 (10.9)	5 (9.1)	8 (14.5)
GDM group	62	5 (8.1)	3 (4.8)	1 (1.6)	2 (3.2)	2 (3.2)
Control group	50	2 (4.0)	1 (2.0)	0 (0)	1 (2.0)	0 (0)
*χ* ^2^		8.316	4.092	6.500	3.210	8.667
*P*		<0.05^∗^	<0.05^∗^	<0.05^∗^	<0.05^∗^	<0.05^∗^

PGDM; pregestational diabetes mellitus; GDM: gestational diabetes mellitus.

## Data Availability

The datasets during the current study are available from the corresponding author on reasonable request.
